# Mechanical Analysis of Posterior Pedicle Screw System Placement and Internal Fixation in the Treatment of Lumbar Fractures

**DOI:** 10.1155/2022/6497754

**Published:** 2022-04-11

**Authors:** Shengkai Mu, Jingxu Wang, Shuyi Gong

**Affiliations:** Shenyang Orthopedic Hospital, Shenyang, Liaoning 110044, China

## Abstract

**Objective:**

Image segmentation technology is applied to separate a single vertebra from the three-dimensional model of the spine, so as to separate a single vertebra image with smaller error, higher degree of automation, and better results. The objectives are to study the biomechanical characteristics of posterior short-segment pedicle screw fixation by three-dimensional finite element method, analyze the mechanical characteristics of posterior pedicle screw rod fixation system under different factors, and demonstrate the feasibility of its application in the treatment of lumbar fracture.

**Methods:**

The authors searched the database for articles about the treatment of lumbar spine fracture, screw rod internal fixation system, and its mechanical parameters. The threshold segmentation method based on region segmentation method was used to segment the image, and the three-dimensional finite element model was used to analyze the biomechanical characteristics of different posterior internal fixation for lumbar spine fracture.

**Results:**

The posterior pedicle internal fixation system for the treatment of multilevel spinal fractures is a mature surgical technique and has fewer postoperative complications. Transpedicle fixation is effective and reliable. It can effectively restore the coronal and sagittal curvature of the vertebral body and restore the stability of the spine better. But the choice of internal fixation method should be individualized based on fracture type, identification of critical and secondary injury sites, and stability assessment. Only after mastering the biomechanical characteristics of the posterior screw rod system for the treatment of lumbar fracture, selecting the appropriate method, and fixing the appropriate movement unit can the best fixation be achieved.

**Conclusion:**

Threshold method is the most direct and simple image segmentation method. The core technology of thresholding is the selection of threshold, which will affect the final segmentation effect. The most common segmentation method is to calculate the segmentation threshold by histogram. The threshold method has less computation and good segmentation effect for the image with large contrast between background and target. Posterior pedicle screw rod system internal fixation has the advantages of less trauma, good reduction, reliable fixation, and less complications. The design, placement angle and depth of various internal fixation systems, and the number of fixed segments all show different mechanical characteristics. As long as we master the above characteristics, choose the appropriate method and fix the appropriate motor unit, and we can get the best fixation; it can be used as an effective treatment for lumbar fracture.

## 1. Introduction

Spinal fractures are not uncommon, and various types of spinal fractures have become a common orthopedic injury. In various kinds of spinal fractures, lumbar fractures have become a common and high incidence of spinal fracture due to their special anatomical and mechanical characteristics [1]. The spinal lumbar segment consists of five vertebrae, two adjacent vertebrae and the disc, joint protrusion, and ligament structures that connect them are known as the spinal function unit, also known as the movement segment. FSU is the smallest unit that can reflect the biological characteristics of the spine, and it is also the most basic unit for maintaining the stability of the spine [2]. The stability of the lumbar spine is the equilibrium state when the endogenous stabilizing factors of the motion segment interact with the external load. Lumbar spine fractures are mostly caused by direct or indirect violence, and the patients are accompanied by local pain and swelling. Lumbar spine fracture surgery is divided into anterior and posterior approaches, as well as long- and short-segment fixation methods. Most factors that cause spinal stenosis come from the front. The anterior decompression is relatively complete, but the posterior internal fixation is more clearly exposed, and the internal fixation is more reliable.

The finite element method was proposed in 1943 to analyze the torsion gastric body, and then, it was applied in the design of aircraft and developed into the matrix displacement method. With the development of computer technology and software technology, the finite element method has also been continuously developed, from solid mechanics to biomechanics, fluid mechanics, magnetic and temperature fields, and other fields. In the field of biomechanics, it can be used to establish a three-dimensional finite element simulation model of the human body and perform corresponding stress and modal analysis on it. It is widely used in the analysis of biomechanics in the field of orthopedics [3]. The finite element method can simulate the mechanical changes of the spine by establishing a spine model and is a reasonable and effective tool in the study of spine mechanics [4]. This article uses three-dimensional finite element method to establish a lumbar fracture internal fixation model, conducts finite element analysis on the biomechanical characteristics of the injured vertebral body, and explores the posterior single-segment fixation and conventional short-segment fixation of the lumbar spine fracture. The biomechanical characteristics provide a basis for the choice of internal fixation for thoracolumbar fractures in clinical practice.

## 2. Materials and Methods

### 2.1. Vertebra Separation Based on Image Segmentation Method

Image segmentation refers to distinguishing different regions with special meanings in an image. These regions do not cross each other, and each region meets the consistency of a specific region. The features available for image segmentation include the following: image grayscale, color, texture, local statistical features, or spectral features. The difference in these features can be used to distinguish different target objects in the image. Medical image segmentation is to distinguish different regions with special anatomical functions in medical images, and each region meets regional consistency. Based on the threshold segmentation method in the area segmentation method, the image can be effectively segmented when the gray value or other characteristic values of different types of objects are very different [5]. The method of threshold segmentation is divided into single threshold segmentation and multithreshold segmentation. As we all know, there are large grayscale differences between bones and muscles, skin, and other soft tissues in CT images. For this reason, this article uses only a single threshold to segment bone images from the original data, that is, the tissue whose gray value is greater than the set threshold is the bone [6–8].

Let (*fi*, *j*) be the gray value of the pixel (*i*, *j*), and the binarization process can be carried out according to formula (1). Among them, *T* is the threshold of binarization, and the gray level of the image is 0~*N*.

(1) $$\begin{array}{c} f\left(i,j\right)=\left\{\begin{array}{cc} N & f\left(i,j\right)\geq T,\\ 0 & f\left(i,j\right)<T. \end{array}\right. \end{array}$$

Figure 1 shows the gray value histogram of any one of the CT slice images of the spine. It can be seen from the histogram that the peak value of the maximum gray value is concentrated between the gray levels of 1170 to 1230. In the experiment, set the gray threshold to 1200. The effect before and after threshold segmentation is shown in Figures 2(a) and 2(b).

The lesion area will produce many isolated small dots and holes, and cracks will appear between the contour lines, as shown in Figure 2(b). In order to solve these problems, the method of mathematical morphology is introduced for filtering. Mathematical morphology image processing includes four basic operations or operations: dilation, erosion, opening, and closing. The experiment mainly adopts the opening operation (opening), that is, the process of corrosion first and then expansion. This operation can eliminate outliers, small objects, separate objects with fine points, and smooth large boundaries without significantly changing the target area. Its definition is shown in formula (2).

(2) $$\begin{array}{c} A\circ B=\left(A\Theta B\right)⊕B. \end{array}$$

In general, continuous opening operations can significantly improve the phenomenon of unsmooth target boundaries, small holes in the target area, and isolated noise in the background area in the image after the binarization operation.  Figure 3 is the result of the opening operation. Compared with Figure 2(b), the scattered points, burrs, and small bridges in the original Figure 2(b) have been cleanly removed.

Perform noise removal on the original noisy CT image, perform a single threshold combined with morphological segmentation on the CT image, and retain only the spine part of the figure; perform three-dimensional reconstruction of the segmented results to obtain a three-dimensional model of the entire spine; use spatial superneighbors. Use domain algorithm to separate individual vertebra from the three-dimensional model of the spine, shown in Figure 4.

In response to the needs of virtual spine correction surgery, the research proposed a general process for processing CT image slice preprocessing. At the same time, according to the spatial superneighborhood algorithm, each single vertebra was automatically separated, and the separated single vertebra was in phase with the original vertebra. The ratio error is smaller, the degree of automation is higher, and the result is ideal. It has certain guiding significance for virtual spine correction surgery. It can be used for three-dimensional reconstruction of tissues and organs, medical image analysis, and the formulation of improved spine surgery plans.

### 2.2. Establishment of a Three-Dimensional Finite Element Model of Normal Thoracolumbar Spine and Fractures

Young male volunteers were selected, and X-ray films were taken before data acquisition to rule out pathological conditions of the spine. Use GE's LightSpeed 16-slice spiral CT to scan the spine T10~L2 continuously along the cross section. The scanning conditions are as follows: the scanning voltage is 120 kV, the scanning current is 300 mA, the layer thickness is 1.25 mm, and the layer interval is 0.625 mm. The scanned CT images are stored in the Dicom3.0 standard. The abovementioned CT data in Dicom format was imported into Mimics 10.01 (Materialise, Belgium), and the three-dimensional model of the spine T10~L2 was established through operations such as threshold segmentation, dynamic area growth, and three-dimensional calculation, and the reverse engineering software Geomagic Studio was used for smooth processing. The finite element preprocessing software Hypermesh was used to supplement the establishment of intervertebral discs and corresponding ligaments. The area of the nucleus pulposus was about 43% of the total area of the intervertebral disc. The annulus fibrosus was simulated as a matrix containing fibers arranged obliquely 30°. Divide each part of the mesh and assign different material properties. Establish a normal model of T10~L2 segment. According to Denis spine fracture classification, a model of incomplete fracture of the upper part of the T12 vertebra was established [9–12]. The specific settings are as follows: remove the upper 1/2 cortical bone of the anterior middle part of the T12 vertebral body, and give the upper endplate and the upper 1/2 cancellous bone material properties of the anterior middle part after injury, shown in Figure 5.

### 2.3. Establishment of Three-Dimensional Finite Element Model of Single-Segment Fixation and Conventional Short-Segment Fixation through Injured Vertebra

Use the Pro/Engineer software to three-dimensionally reconstruct the internal fixation system used in spinal lumbar fracture surgery, and assemble it with the three-dimensional model of the spine from T10 to L2. Among them, due to the fracture of the upper part of the T12 vertebral body, the T11 and T12 vertebral bodies were fixed by a single-segment fixation model of the injured vertebra. The conventional short-segment internal fixation model fixes the T11 and L1 vertebral bodies across the segments. The screw placement and fixation methods refer to literature. The models of single-segment fixation and conventional short-segment fixation through injured vertebrae are shown in Figure 6.

A finite element analysis of transtraumatic and transtraumatic screw placement showed that transtraumatic screw placement was more effective in alleviating postoperative pain and improving spinal stability in the short and long term, although the operative time was longer and there was more intraoperative bleeding. In addition, transtraumatic screw placement may result in a lower rate of internal fixation failure.

### 2.4. Posterior Pedicle Screw System Internal Fixation for the Treatment of Lumbar Fractures

Pedicle internal fixation is suitable for patients with various unstable fractures and dislocations of the thoracolumbar spine or paraplegia: patients with spinal deformities, such as intervertebral disc degeneration, lumbar spondylolisthesis, and kyphosis. Dorsal midline incision is made with the diseased spine as the center, the position and direction of the pedicle screw are determined, the pedicle screw is inserted, the internal fixation device is placed, and the pedicle screw is reduced and fixed, as shown in Table 1.

The pedicle screw is a short-segment internal fixation system with superior biomechanical properties. Studies have shown that a posterior short-segment pedicle screw can transmit corrective forces to the three spinal columns through the posterior approach to the anterior part of the vertebral body. It is a mechanical tension fix with 6 degrees of freedom in three-dimensional space. Correct deformities and reduce fractures. The front, middle, and rear columns can be fixed at the same time. Effective anatomical reduction can be achieved even for difficult-to-reduce fractures. In addition, the feature of short-segment fixation avoids the impact of long-segment fixation on mobility and complications such as chronic low back pain and “flat back deformity.” Effectively preserving motion segments can provide immediate stabilization of the spine, reduce the chance of nerve damage, and be safer and more reliable. Preoperative X-ray, CT or MRI examination can comprehensively evaluate and understand the fracture site, degree, type, spinal cord compression, attachment fracture, etc., and determine the method and scope of decompression.

After a lumbar fracture, the stability of the spine is destroyed and often accompanied by spinal cord nerve injury. The main factors that cause the spinal nerve compression are the bone mass behind the vertebral body and the compression of the upper edge of the injured vertebra due to the kyphosis angle and the displacement between the vertebral bodies [13]. The purpose of surgical treatment of lumbar fractures is to reconstruct the shape of the spinal canal, restore the stability of the spine, and eliminate the compression on the spinal cord. Restore the effective volume and stability of the spinal canal, and relieve the nerve compression in a timely and complete manner, which is conducive to the recovery of spinal nerve function. Removal of compressive material in front of the spinal cord, adequate decompression of the spinal canal, correction of deformities, reconstruction of spinal stability, and bone graft fusion have been recognized by most scholars. Thirty-five cases of thoracolumbar fractures were treated with posterior pedicle screw system internal fixation, of which 20 cases underwent intraoperative posterior decompression, and 8 cases underwent bone grafting of the diseased vertebrae through the pedicle. All 35 cases underwent bone grafting between the articular and transverse processes, and the average height (percentage) of the anterior and posterior edges of the injured vertebrae before and after the operation, the Cobb's angle, and the cross-sectional area of the spinal canal were measured. 35 cases of lumbar fractures were treated with posterior spinal canal decompression and nail-rod system internal fixation, and satisfactory results were achieved, as shown in Figure 7.

### 2.5. Mechanical Experimental Study of Lumbar Internal Fixation

In 1988, Gurr et al. [14] compared the fixation effect of the Kaneda system with pedicle screws on the calf spine, and the results showed that the effect of the former fixation of 3 segments is equivalent to that of the latter fixation of 5 segments. Zdeblick et al. [15] and An et al. [16] compared several anterior internal fixation devices and found that the Kaneda system had the best stability. An et al. [17] proved through experiments that the use of a nut that prevents the screw from exiting will greatly enhance the fixing strength of the anterior internal fixation system. The posterior internal fixation system mainly includes pedicle screw and hook rod system. It is generally believed that the stiffness of the former is significantly higher than that of the latter. Lim et al. [18] confirmed through experiments that the axial torsional stability of the pedicle screw system is enhanced after the use of the transverse connecting rod, but the stability does not change significantly when subjected to other types of loads. Lynn et al. [19] found that the use of two transverse connecting rods can significantly increase the rotational and bending stiffness. There have been some studies on the pullout strength of pedicle screws. It is generally believed that the diameter of the pedicle screw is the most important factor. The larger the diameter of the screw, the higher the pullout strength. Another important factor that affects the strength of pedicle screw extraction is the shear strength of the pedicle and vertebral body, which is mainly related to the bone density of the cancellous bone and the torque when the screw is inserted. The lower the bone density, the lower the pull-out strength of the screw. Therefore, when the pedicle screw is located in an area with high bone density near the endplate, its extraction strength is relatively high. In the past, we mostly paid attention to the stability of the spine itself, ignoring the load-bearing effect of the internal fixation. When the fatigue strength of the internal fixation is lower than the breaking strength, it is necessary to effectively reduce the stress of the internal fixation. Cunningham et al. [20] used 12 kinds of pedicle screws to fix the vertebral body in the biomechanical experiment and found that the compressive strength and bending strength of all specimens were significantly lower than normal. It can be seen that if the stability of the anterior structure cannot be effectively reconstructed, the pedicle screw system will bear part or even all of the load originally borne by the anterior column. Clinical reports about broken nails and implant loosening after the treatment of thoracolumbar vertebral fractures with posterior pedicle screw system are not uncommon, most of which are cases of continuous damage to the anterior column, and if anterior bone grafting is performed at the same time, no such complications occurred. Cripton et al. [21] analyzed the load-sharing effect of the posterior lumbar internal fixation system and believed that the risk of damage to the posterior internal fixation system is great when severe anterior injury occurs, as shown in Figures 8 and 9.

## 3. Results

Biomechanical studies have shown that the posterior pedicle short-segment fixation has a firm three-column fixation function, which is a tension fixation in terms of spine mechanics. The short-segment pedicle internal fixation system can reconstruct the stability of the spine, restore the volume of the spinal canal, and provide a favorable external environment for the recovery of nerve damage. Fracture reduction is divided into direct reduction and indirect reduction. When the posterior screw rod is stretched longitudinally to restore the height of the spine and the posterior column, the posterior longitudinal ligament is stretched to achieve indirect reduction of the bone block in the spinal canal, and the rod is used for prereduction. Bent, angled pedicle screws and the lever force of expansion can restore the height of the anterior column. Whether it is a compression or burst fracture, as long as the anterior and posterior longitudinal ligaments are intact, most of the fracture fragments can be reduced satisfactorily through the expansion of the AF internal fixation system. During the operation, the fractured vertebrae should be determined under X-ray fluoroscopy, and the position, direction, depth, and reduction of the screw should be observed to prevent poor reduction and excessive expansion. When determining the position of the guide pin of the pedicle screw, the standard positive and lateral X-ray film is used to determine the position of the guide pin. If the positions of the screws on both sides are not symmetrical, the stresses received by the rod structures on both sides will be different, leading to complications such as bent or broken nails after surgery [22]. According to the patient's symptoms and signs, as well as the extent and extent of the kyphosis of the fracture, and the location and extent of spinal cord compression provided by the patient, select the decompression method and decompression range. Most of the posterior longitudinal ligaments with small fractures in the spinal canal are intact. Most of the fractures can be automatically reset by the force of expansion; for those with large fractures in the spinal canal that cannot be indirectly reset, the semilaminar or full-laminectomy is used. The blunt-head chisel strikes forward carefully to hit the fractured piece directly into the vertebral body to achieve the purpose of decompression. For large fractures in the spinal canal and obvious stenosis of the spinal canal, especially in patients with burst fractures of the lumbar spine, the anterior and posterior longitudinal ligaments have been damaged in most cases. Resection of the medial semi cortex and part of the facet joints of one or both sides of the pedicle, and then, decompress after reaching the front of the spinal canal; after distraction, the vertebral body of the injured vertebral body has the phenomenon of “hollow vertebral body” or cannot achieve distraction reduction. The anterior and middle columns lose their structural integrity. Without effective bone grafting, internal fixation fatigue, fracture, and collapse of the fractured vertebral body and loss of correction may occur in the late stage. Parker et al. [23] believe that the failure rate of internal fixation devices can reach 9% to 54% if only posterior fixation of burst fractures of the lumbar spine, without the support of the anterior column. Therefore, during the operation, it is necessary to focus on the decompression of the front of the spinal canal, as well as the recovery of the height of the diseased vertebrae and the bone mass. Therefore, we take the iliac bone from the body and implant the diseased vertebral body through the pedicle to restore its height as much as possible. At the same time, the lamina and spinous process removed during the operation are bitten into granules and placed on the transverse process and the small joints on the unopened side. Bone grafting was performed between the processes to achieve the purpose of spine stabilization. For the free bone fragments and intervertebral disc tissues in the spinal canal, all need to be removed with a small curette or nucleus pulposus forceps, fully decompressed, and at the same time, carefully protect the spinal nerve with nerve stripping paper.

At present, the clinical treatment of lumbar spine fractures mostly uses posterior pedicle screw internal fixation, which is beneficial to the recovery of lumbar spine function as soon as possible. With the increasing understanding of the pathogenesis of spinal fractures, there is an urgent need for systematic and comprehensive biomechanical research on the spine. More and more scholars use the finite element analysis method to analyze the force of the spine under various loads. This method of biomechanical research through the finite element model is indispensable in the study of the biological characteristics of the spine. The important role of substitution not only provides strong guidance for the clinically carried out surgical internal fixation technology but also provides a scientific basis for the evaluation of surgical effects.

## 4. Discussion

### 4.1. The Rear Road Nail Bar System and the Front Road Cone Steel Plate System

Compared with the anterior vertebral plate system, the posterior screw and rod system has obvious mechanical advantages. The screw rod system firmly fixes the pedicle screw and the metal rod through a universal joint and can be adjusted in three dimensions in space, so as to achieve effective reduction and firm fixation of spinal fractures. The nail-rod system has the following characteristics: ① it has a long rod, which can fix longer segments and can fix multiple segments at the same time, which has obvious advantages in treating multisegment fractures; ② it can perform rod pretreatment according to the degree of fracture kyphosis. Bending can meet the correction requirements of different degrees and directions, but because the two rods are prone to asymmetry in the bending, the instability of the rotation direction is easy to occur; ③ it has irreplaceable advantages in spinal correction. AF is usually used for the fixation of single-segment vertebral fractures. For multisegment vertebral fractures, especially skip fractures, the application of AF is limited. The nail-rod combined pedicle internal fixation device can three-dimensionally correct multilateral fractures and displacements of the vertebral body through the expansion and rotation of the instrument. Especially for burst fractures of the vertebral body, it can effectively restore the height of the compressed vertebral body and fix the joints. The segment is short and reliable, in line with the principle of three-dimensional fixation of spinal fractures, shown in Table 2.

With the development of internal fixation devices, pedicle screws can provide better fixation than the first posterior internal fixation devices such as Harrington rods and spinous process plates. In addition, posterior surgery has the advantages of simple operation and less trauma. Posterior pedicle screw internal fixation has become the most widely used surgical method for the treatment of thoracolumbar fractures in clinical practice, but some scholars [24] believe that this approach is more prone to kyphotic deformity compared with anterior surgery loss. Therefore, the selection of the surgical approach should be a reasonable choice by considering factors such as the type, location, nerve injury, and the skill and experience of the surgical operator (Figures 10 and 11).

### 4.2. Posterior Short-Segment and Single-Segment Pedicle Screw Internal Fixation

With the application of posterior short-segment transinjured vertebral nail placement in the treatment of lumbar fractures, some scholars have proposed posterior single-segment pedicle screw instrumentation (MPSI) in order to further reduce the number of fixed segments. For the treatment of thoracolumbar fractures, posterior single-segment pedicle screw internal fixation refers to the focus of the injured vertebrae and adjacent vertebral body segments. It is a development based on the placement of nails in the injured vertebrae. This surgical method mainly relies on a complete endplate. The residual bone on the side stretches the injured vertebrae to restore the original height and fix it. In clinical work, there is also a stabilization effect by only fixing the injured vertebrae and an adjacent normal vertebral body. The concept of fixing only one motion segment is different from the cross-segment pedicle screw internal fixation. McLain et al. [25] found that compared with short-segment fixation, it has the following advantages: one less fusion of the intervertebral space, which can maximize the preservation of the motion segment of the spine; the screw directly screwed into the injured vertebra can immediately open the injured vertebra, to better recover and maintain the height of the injured vertebral; because there are few fixed and fused segments, the degeneration of adjacent segments is reduced, and the postoperative vertebral body instability and loss of correction are minimized; to avoid long-term fixation of the contralateral intervertebral space and reduce regression Change; after posterior pedicle screw fixation, due to the stress shielding effect, most of the stress is transmitted through the posterior column screw. After single-segment fixation, the column torque is reduced, which can reduce the nail-rod stress load and reduce the probability of internal fixation damage. It can also reduce the rate of postoperative correction loss, especially in the treatment of flexion-traction fractures. The effect is more significant; the operation is small, the surrounding tissue is less peeled, the amount of bleeding is less [26–30], and the surgical trauma is reduced, and in most cases, there is no need to take the iliac bone for bone grafting, which avoids the problem of pain in the bone removal area [31] (Figure 12).

### 4.3. Finite Element Research

The biomechanical properties of the lumbar pedicle screw fixation system were evaluated by the finite element method. The results showed that, compared with the traditional lateral pedicle screw fixation system with connecting device, the pedicle screw fixation system with connecting device increased the diagonal direction. It is more stable in flexion and extension; some studies have investigated the force transmission mechanism in the helical bone complex using finite element methods. The results show that the screw is subjected to a series of discrete loads within the vertebral body, resulting in local bending moments. The maximum stress on the screw acts on the screw base and threaded joints, which is consistent with the clinically observed screw fracture sites [32] (Figure 13).

## 5. Conclusion

The posterior pedicle internal fixation system for the treatment of multilevel spinal fractures is a mature surgical technique and has fewer postoperative complications. Transpedicle fixation is effective and reliable. It can effectively restore the coronal and sagittal curvature of the vertebral body and restore the stability of the spine better. But the choice of internal fixation method should be individualized based on fracture type, identification of critical and secondary injury sites, and stability assessment. Only after mastering the biomechanical characteristics of the posterior screw rod system for the treatment of lumbar fracture, selecting the appropriate method, and fixing the appropriate movement unit [33] can the best fixation be achieved.

Image segmentation technology is often used to meet the needs of virtual spine surgery. The commonly used segmentation techniques include “threshold method,” “edge segmentation method,” “region segmentation method,” and some “theory specific segmentation methods.” The threshold method is the most direct and simple method of image segmentation. According to the threshold, the image is divided according to the gray level. But the thresholding method is mainly for gray information, and if the image background is complex or there are multiple targets, it is difficult to ensure the segmentation effect. Threshold segmentation is often used in CT image processing. According to their own experience, doctors constantly adjust the threshold for segmentation until they achieve the desired effect.

## Figures and Tables

**Figure 1:** Example of histogram.

**Figure 2:** Rendering before and after threshold segmentation.

**Figure 3:** Image after opening operation.

**Figure 4:** Single spine model.

**Figure 5:** Three-dimensional model of thoracolumbar T11-L1 segment.

**Figure 6:** 3D finite element fixation models of T10-L2 segment.

**Figure 7:** Finite element model of posterior decompression internal fixation.

**Figure 8:** Anteroposterior and lateral view of finite element model of vertebral fracture.

**Figure 9:** Schematic diagram of simulated pedicle screw placement.

**Figure 10:** Finite element model of normal thoracolumbar vertebral body.

**Figure 11:** Finite element model of anterior internal fixation.

**Figure 12:** Finite element model of spinal T10-L2 segment.

**Figure 13:** Stress nephogram of normal cone in forward and backward flexion.

**Table 1:** Characteristics of pedicle internal fixation system.

Characteristics of pedicle internal fixation system	
Feature 1	Early reduction and internal fixation, fixed tightly
Feature 2	Short-segment fixation
Feature 3	Restore the normal physiological radian of the spine
Feature 4	Restore the cross-sectional area of the spinal canal, rebuild the stability of the spine, achieve effective and complete decompression, and relieve the strain on the spinal nerves. Promote the recovery of nerve function
Feature 5	Full bone graft fusion, high fusion rate of bone graft
Feature 6	Patients can get out of bed early

**Table 2:** The changes of Cobb angle before and after operation were compared between the two groups.

Group	Preoperative	Postoperative	After 1 year
Anterior	25.1 ± 8.9	3.4 ± 1.7	4.6 ± 1.6
Posterior	23.7 ± 7.6	3.2 ± 1.4	8.2 ± 2.1
*T* value	0.757	0.574	9.343
*P* value	0.452	0.567	0.001

## Data Availability

The image data used to support the findings of this study have been deposited in the VerSe 2019 dataset (https://osf.io/nqjyw/).
